The article "Systematic analyses reveal long non-coding RNA (PTAF)-mediated promotion of EMT and invasion-metastasis in serous ovarian cancer" was retracted in 2023. Reasons: duplicated images; unreliable results or conclusions.

# Systematic analyses reveal long non-coding RNA (PTAF)-mediated promotion of EMT and invasion-metastasis in serous ovarian cancer

**DOI:** 10.1186/s12943-018-0844-7

**Published:** 2018-06-21

**Authors:** Haihai Liang, Xiaoguang Zhao, Chengyu Wang, Jian Sun, Yingzhun Chen, Guoyuan Wang, Lei Fang, Rui Yang, Mengxue Yu, Yunyan Gu, Hongli Shan

**Affiliations:** 1 Department of Pharmacology (State-Province Key Laboratories of Biomedicine-Pharmaceutics of China, Key Laboratory of Cardiovascular Research, Ministry of Education), College of Pharmacy, Harbin Medical University, Translational Medicine Research and Cooperation Center of Northern China, Heilongjiang Academy of Medical Sciences, Harbin, 150081 China; 2 Department of Systems Biology, College of Bioinformatics Science and Technology, Harbin Medical University, Harbin, 150001 China; 3 Department of Pathology of The Second Affiliated Hospital, Harbin Medical University, Harbin, 150081 China; 4 Department of Pathology of The First Affiliated Hospital, Harbin Medical University, Harbin, 150081 China; 5 Department of Obstetrics and Gynecology, The Second Affiliated Hospital of Harbin Medical University, Harbin, 150081 China; 6 Department of Systems Biology, College of Bioinformatics Science and Technology, Harbin Medical University, Harbin, 150086 China; 7 Training Center for Students Innovation and Entrepreneurship Education, Harbin Medical University, Harbin, 150086 China

**Keywords:** Serous ovarian cancer, Epithelial-mesenchymal transition, Long non-coding RNA, Invasion, Metastasis

## Abstract

**Background:**

A deeper mechanistic understanding of epithelial-to-mesenchymal transition (EMT) regulation is needed to improve current anti-metastasis strategies in ovarian cancer (OvCa). This study was designed to investigate the role of lncRNAs in EMT regulation during process of invasion-metastasis in serous OvCa to improve current anti-metastasis strategies for OvCa.

**Methods:**

We systematically analyzes high-throughput gene expression profiles of both lncRNAs and protein-coding genes in OvCa samples with integrated epithelial (iE) subtype and integrated mesenchymal (iM) subtype labels. Mouse models, cytobiology, molecular biology assays and clinical samples were performed to elucidate the function and underlying mechanisms of lncRNA PTAF-mediated promotion of EMT and invasion-metastasis in serous OvCa.

**Results:**

We constructed a lncRNA-mediated competing endogenous RNA (ceRNA) regulatory network that affects the expression of many EMT-related protein-coding genes in mesenchymal OvCa. Using a combination of in vitro and in vivo studies, we provided evidence that the lncRNA PTAF-miR-25-SNAI2 axis controlled EMT in OvCa. Our results revealed that up-regulated PTAF induced elevated SNAI2 expression by competitively binding to miR-25, which in turn promoted OvCa cell EMT and invasion. Moreover, we found that silencing of PTAF inhibited tumor progression and metastasis in an orthotopic mouse model of OvCa. We then observed a significant correlation between PTAF expression and EMT markers in OvCa patients.

The article "Systematic analyses reveal long non-coding RNA (PTAF)-mediated promotion of EMT and invasion-metastasis in serous ovarian cancer" was retracted in 2023. Reasons: duplicated images; unreliable results or conclusions.

**Conclusions:**

The lncRNA PTAF, a mediator of TGF-β signaling, can predispose OvCa patients to metastases and may serve as a potential target for anti-metastatic therapies for mesenchymal OvCa patients.

**Electronic supplementary material:**

The online version of this article (10.1186/s12943-018-0844-7) contains supplementary material, which is available to authorized users.

## Background

Ovarian cancer (OvCa) is one of the most lethal malignancies in women worldwide. The high mortality rate of OvCa patients is due primarily to direct invasion of adjacent organs or metastasis to the peritoneal cavity [1]. However, the underlying molecular mechanisms that mediate OvCa cell metastasis remain largely unclear. Elucidating the mechanism involved in the invasion or metastasis of OvCa cells may promote the development of effective metastasis-targeted therapies and improve the overall survival of OvCa patients [2].

Epithelial-to-mesenchymal transition (EMT) is characterized by the loss of cell-cell adhesions and gain of migratory and invasive traits; this process governs events such as embryonic development, tissue regeneration, organ fibrosis, and tumor cell metastasis [3–5]. The transforming growth factor (TGF)-β signaling pathway is a major inducer of EMT and promotes breast cancer metastasis [6]. In addition to TGF-β, several other tyrosine kinase receptors, such as insulin-like growth factor and platelet-derived growth factor, also play critical roles in regulating EMT during tumor progression [7]. These inducers converge on the activation of one or more transcription factors (TFs), including SNAI1, SNAI2, ZEB1, ZEB2, TWIST1 and TWIST2, that directly or indirectly repress the E-cadherin (CDH1) promoter [8]. The inactivation of E-cadherin is considered a hallmark of EMT. EMT has been shown to play a critical role in cancer cell metastatic dissemination events by endowing cancer cells with a more motile and invasive phenotype [9]. Emerging evidence suggests that the acquisition of invasiveness in OvCa cells is accompanied by the loss of epithelial features and gain of a mesenchymal phenotype, also known as EMT [10]. However, the molecular events that drive the EMT process during OvCa progression are largely unknown [11].

MicroRNAs (miRNAs) are a class of small non-coding RNAs approximately 22 nucleotides in length that regulate the gene expression of their targets by triggering mRNA degradation or protein translation inhibition [12]. Several miRNAs, such as miR-200 family members, have been found to regulate EMT by targeting the E-cadherin repressors ZEB1 and ZEB2 [13, 14]. Yang et al. identified a miRNA regulatory network in mesenchymal OvCa [1]. The network consists of 8 major miRNAs (miR-25, miR-506, miR-29c, miR-182, miR-128, miR-101, miR-141, and miR-200a), among which miR-141, miR-200a, miR-101 and miR-506 have been reported to be regulators of EMT [1, 13, 15]. Long non-coding RNAs (lncRNAs) are a class of transcripts longer than 200 nucleotides with no protein coding potential. Dysregulated lncRNA expression is frequently reported in different cancer types and is correlated with cancer aggressiveness. Overexpression of the lncRNAs HOTAIR and HOXA11 has pro-metastatic effects on OvCa cells, and these effects were shown to be partially mediated by EMT-related genes [16, 17]. LncRNAs could function as miRNA sponges and act as competing endogenous RNAs (ceRNAs), competitively binding to miRNAs to affect the expression level of protein-coding genes [18]. However, currently, the functional significance and targets of these lncRNA-mediated EMT regulation mechanisms in OvCa are mostly unknown.

The article "Systematic analyses reveal long non-coding RNA (PTAF)-mediated promotion of EMT and invasion-metastasis in serous ovarian cancer" was retracted in 2023. Reasons: duplicated images; unreliable results or conclusions.

Thus, a deep understanding of the molecular regulatory mechanisms of EMT involving lncRNAs, TFs and miRNAs during OvCa invasion is urgently needed. In this study, we used an integrative approach and analyzed multi-dimensional data from 459 serous OvCa cases in The Cancer Genome Atlas (TCGA) to uncover the underlying molecular network of the mesenchymal OvCa subtype. We constructed a ceRNA regulatory network for mesenchymal OvCa and focused on the role of PTAF-miR-25-SNAI2 in TGF-β-induced EMT and in the invasion-metastasis cascade of OvCa.

## Methods

### Data collection and processing

As shown in the flowchart in Fig. 1a, we collected two sets of mRNA and lncRNA OvCa expression data from TCGA and GSE9891 from the Gene Expression Omnibus, both of which had integrated epithelial (iE) subtype and integrated mesenchymal (iM) subtype labels [1]. The level 3 gene expression data from TCGA were used in this work. The processed sequencing expression profiles of lncRNAs in the TCGA OvCa dataset were obtained in The Atlas of Non-coding RNAs in Cancer (TANRIC) database [19]. The lncRNAs with non-zero expression in at least 80% of the samples were retained. The lncRNA expression profile of the GSE9891 dataset was re-annotated using the Affymetrix Human Genome U133 Plus 2.0 Array (HG-U133 Plus 2.0). The detailed method of re-annotation were presented in [20]. If multiple probe-sets were mapped to the same lncRNA, the expression value of the lncRNA was summarized as the mean of the values of multiple probe-sets. Agilent Human miRNA Microarray data for OvCa and normal samples were obtained from TCGA. The data are summarized in Additional file 1: Table S1.

The article "Systematic analyses reveal long non-coding RNA (PTAF)-mediated promotion of EMT and invasion-metastasis in serous ovarian cancer" was retracted in 2023. Reasons: duplicated images; unreliable results or conclusions.

**Fig. 1:** Identification of the EMT-related ceRNA regulatory network. **a** Flowchart of the integrative analysis. **b** The ceRNA network in mesenchymal OvCa. Rounded rectangles, ellipses and hexagons denote lncRNAs, EMT genes and miRNAs, respectively. The lncRNAs and EMT genes, which are shown in blue, were significantly up-regulated in mesenchymal OvCa compared with epithelial OvCa. Up-regulated miRNAs are shown in red, and down-regulated miRNAs are shown in green. **c** Genomic distance between lncRNAs and correlated EMT genes. SNAI2 was significantly up-regulated in mesenchymal OvCa compared with epithelial OvCa in the TCGA (**d**) and GSE9891 (**e**) data sets. Kaplan-Meier overall survival curves for OvCa patients with high and low expression of SNAI2 in the TCGA (**f**) and GSE9891 (**g**) data sets. **h** miR-25 was significantly down-regulated in mesenchymal OvCa compared with epithelial OvCa in the TCGA data set. The lncRNA PTAF was significantly up-regulated in mesenchymal OvCa compared with epithelial OvCa in the TCGA (**i**) and GSE9891 (**j**) data sets

Three hundred and seventy-seven EMT-related genes were downloaded from dbEMT (http://dbemt.bioinfo-minzhao.org/) [21]. The miRNA-mRNA interactions, which were recorded in at least two of the databases of TargetScan [22], miRanda [23], miRBase [24] and miRTarBase [25], were included in our analysis. The miRNA-lncRNA interactions were collected from databases of starBase [26] and miRcode [27].

### Identification of mesenchymal-related ceRNAs

To identify differentially expressed (DE) genes, lncRNAs and miRNAs in the iM subtype compared with the iE subtype of OvCa, t tests were performed, and the *P* values were corrected using the Benjamini-Hochberg method. Pearson’s correlation test was used to calculate the correlation between the expression of DE genes and DE lncRNAs. A hypergeometric distribution model was used to test whether the DE EMT genes shared a significant number of miRNA binding sites with DE lncRNAs. The mesenchymal-related ceRNAs were selected according to the following criteria: (1) The DE EMT genes (DE lncRNAs) were consistently differentially expressed in both data sets and with the same dysregulation direction under the constraint of a false discovery rate (FDR) < 0.1. (2) The expression of DE EMT genes and DE lncRNAs was significantly correlated (*P* < 0.05 and *r* ≥ 0.4) and they bound to a significant number of common miRNAs (*P* < 0.05). The ceRNA network was presented using the Cytoscape web tool (http://js.cytoscape.org). All analysis processes were performed in R 3.2.3 (https://www.r-project.org/).

The article "Systematic analyses reveal long non-coding RNA (PTAF)-mediated promotion of EMT and invasion-metastasis in serous ovarian cancer" was retracted in 2023. Reasons: duplicated images; unreliable results or conclusions.

### Clinical samples and in situ hybridization

Forty-nine formalin-fixed, paraffin-embedded serous OvCa tissue samples from the Second Affiliated Hospital of Harbin Medical University were collected for in situ hybridization (ISH) analysis. All experiments were approved by the Ethics Committee of Harbin Medical University. ISH was performed as previously described [1]. Briefly, 4-μm-thick tissue sections were deparaffinized in xylene and dehydrated in an ethanol dilution series. The slides were submerged in diethylpyrocarbonate–treated water and subjected to proteinase K digestion (5–10 μg/mL) and 0.2% glycine treatment, refixed in 4% paraformaldehyde, and treated with acetylation solution [66 mmol/L HCl, 0.66% (*v*/v) acetic anhydride, and 1.5% (v/v) triethanolamine]. The tissues were pre-hybridized for 1 h at 37 °C and then hybridized with a digoxigenin (DIG)-labeled PTAF-specific probe (5’-TGGGC CATAA GAGTG AAACT CCATC CACGT TTGTG GTCTG-3′) overnight at 37 °C. The next day, the tissues were washed as follows: 2X SSC for 10 min at 37 °C, 1X SSC for 5 min twice at 37 °C, and 0.5X SSC for 10 min at room temperature. The sections were blocked with BSA for 30 min, and the DIG label was detected with a polyclonal anti-DIG antibody and an alkaline phosphatase-conjugated secondary antibody (Ventana), using NBT/BCIP as the substrate.

Signals in tumor cells were visually quantified using a scoring system from 0 to 9, and the score was determined by multiplying the signal intensity by the percentage of positive cells (signal: 0 = no signal, 1 = weak signal, 2 = intermediate signal, and 3 = strong signal; percentage: 0 = 0%, 1 ≤ 25%, 2 = 25–50%, and 3 ≥ 50%).

### Cell culture and treatment

SKOV3, A2780 and OVCAR-3 cells were purchased from the Cell Bank of the Chinese Academy of Sciences (Shanghai, China). The cells were grown in 25 cm^2^ cell culture flasks with Dulbecco’s Modified Eagle Medium (DMEM, HyClone) or RPMI 1640 (HyClone) supplemented with 10% fetal bovine serum (FBS, HyClone), 2 mM L-glutamate, 100 U/ml penicillin G, and 100 U/ml streptomycin at 37 °C in 5% CO_2_, 95% air. The cells were maintained at a specific density, and a day before infection, the cells were seeded into 6-, 12- or 24-well culture plates at the appropriate cell density.

### Cell transfection

Prior to transfection, cells were washed with sterile PBS and incubated with serum-free medium for 4–6 h. A miRNA, PTAF or shRNA construct and the transfection reagent were separately mixed with Opti-MEM®I Reduced Serum Medium (Gibco, Grand Island, NY), and the two mixtures were combined and incubated at room temperature for 15 min. The cells were then incubated with the transfection mixture for 6–8 h. Then, fresh medium containing 10% FBS was added to the cell culture plates, and the cells were cultured for the following experiments.

The article "Systematic analyses reveal long non-coding RNA (PTAF)-mediated promotion of EMT and invasion-metastasis in serous ovarian cancer" was retracted in 2023. Reasons: duplicated images; unreliable results or conclusions.

### Western blotting

For western blot analyses, total protein was extracted from SKOV3 cells. The cells were lysed on ice with RIPA lysis buffer (Beyotime, Jiangsu, China) containing protease inhibitors. The protein samples (40 μg) were fractionated on 8% SDS-polyacrylamide gels and transferred onto pure nitrocellulose membranes (Pall Life Science). The membranes were then probed with primary antibodies, and GAPDH was used as an internal control (the anti-GAPDH antibody was purchased from Kangchen, Shanghai, China). Primary antibodies against Vimentin and SNAI2 were purchased from Cell Signaling Technology. The primary antibody against E-cadherin was purchased from Proteintech (Rosemont, IL, USA). The immunoreactive bands were detected using an Odyssey Infrared Imaging System (Gene Company Limited, Hong Kong, China). The intensity of each band was measured with Odyssey 3.0 software.

### Quantitative RT-PCR

Total RNA was extracted from OvCa patient samples, SKOV3 cells or A2780 cells using Trizol (Invitrogen, Carlsbad, CA). As described in our previous work [4], qRT-PCR was performed on a 7500 Fast Real-Time PCR System (Applied Biosystems) using Power SYBR® Green Master Mix (Applied Biosystems). After the reactions were complete, the comparative threshold cycle (Ct) method was used to calculate the relative gene (e.g., miRNA, E-cadherin, vimentin, and SNAI2) expression. GAPDH or U6 was used as an internal control.

### Immunohistochemistry staining

Immunohistochemistry (IHC) analysis was performed as previously described [28]. Clinical tissues from OvCa patients were fixed with 4% paraformaldehyde for 7 days, paraffin-embedded and serially sectioned. Primary antibodies against E-cadherin and SNAI2 were purchased from Proteintech (Rosemont, IL, USA). The staining was analyzed under a fluorescence microscope (DP80, Olympus, Japan).

### Scratch wound-healing assay

To determine the regeneration and repair abilities of OvCa cells, SKOV3 or A2780 cells were seeded in 6-well plates and incubated overnight at 37 °C with 5% CO_2_. Artificial wounds were made using 10-μl pipette tips (0 h) to generate a gap in the confluent cell layer. The cells were washed with PBS and incubated with either serum-free medium as a control or different treatment combinations (miR-25 mimic, negative controls, miR-25 inhibitor, etc.). Phase-contrast images were taken at different time points using a microscope (Nikon TS100, Japan).

The article "Systematic analyses reveal long non-coding RNA (PTAF)-mediated promotion of EMT and invasion-metastasis in serous ovarian cancer" was retracted in 2023. Reasons: duplicated images; unreliable results or conclusions.

### Cell migration and invasion assays

The detailed procedures of the cell migration and invasion assays were described in a previous study [29]. Briefly, 5 × 10^4^–10^5^ cells in serum-free medium were seeded into the upper layer of a Transwell membrane insert with an 8 μm pore size in a 24-well plate (Corning). The membranes were coated with Matrigel (BD Biosciences) for invasion assays or left uncoated for migration assays. Then, medium containing 10% FBS was placed in the bottom chamber as an attractant. After 36 h, the cells were fixed with methanol and stained with crystal violet. The cell numbers were counted using Image-Pro Plus 6.0.

### Generation of stable PTAF knockdown or overexpression cell lines

In accordance with the manufacturer’s instructions, stable PTAF knockdown or overexpression SKOV3 cell lines and respective control cell lines were generated using lentiviral vectors carrying either sh-PTAF, a PTAF overexpression construct, or the respective negative controls (Biowit Technology, Shenzhen, China). Stable cells were selected by treatment with 2 μg/ml puromycin and 200 μg/ml G418. These cell lines were used for experiments in the nude mouse xenograft tumor model described below.

### Xenograft model of ovarian cancer

A xenograft model of OvCa was established using stable SKOV3 cell lines in which the lncRNA PTAF was knocked down (sh-PTAF group) or not (sh-Scramble group) or those in which the PTAF was overexpressed (PTAF group) or not (pcDNA3.1 group). Four- to 6-week-old female BALB/c nude mice were obtained from SLRC Laboratory Animals (Shanghai, China) and randomly divided into four groups (*n* = 10 for each group). Approximately 1 × 10^6^ cells were injected into the nude mice through an intraperitoneal injection. After 4 weeks, all mice were sacrificed, and the tumor tissues were dissected. In addition, the peritoneal nodules were counted, collected, weighed and photographed. For in vivo imaging analysis, BALB/c nude mice were injected intraperitoneally with 10 μl of D-luciferin (15 mg/ml)/g of body weight, and approximately 3 min later, the mice were anesthetized with diethyl ether and imaged using an IVIS Lumina system (Xenogen, Hopkinton, MA).

### Luciferase activity assay

Sequences of the SNAI2 3’UTR or PTAF containing wild-type or mutated miR-25 binding sites were synthesized by Invitrogen and amplified by PCR. The PCR fragments were subcloned into the SacI and HindIII sites downstream of the luciferase gene in the pMIR-Report plasmid (Promega). A miR-25 sensor reporter was constructed according to the method described previously [30] . Briefly, the mouse genomic sequence (200 bp) flanking pre-miR-25 was reversely inserted into the pGL3 vector downstream of the luciferase coding region. Next, the luciferase vector (0.1 μg) was cotransfected with a miR-25 mimic or PTAF into HEK-293 cells or SKOV3 cells using Lipofectamine 2000 (Invitrogen, Carlsbad, CA). As an internal control, 10 ng of a Renilla luciferase reporter vector was also included. After 48 h of transfection, the cells were collected, and the luciferase activities were measured using a luminometer according to the manufacturer’s instructions.

The article "Systematic analyses reveal long non-coding RNA (PTAF)-mediated promotion of EMT and invasion-metastasis in serous ovarian cancer" was retracted in 2023. Reasons: duplicated images; unreliable results or conclusions.

### Pull-down assay with biotin-tagged miRNA

SKOV3 cells were transfected with biotin-tagged miRNA (100 nM) as previously described [31] and harvested 48 h after transfection. The cells were washed with PBS followed by a brief vortex and incubated in lysis buffer on ice for 10 min. The lysates were incubated with M-280 streptavidin magnetic beads (Sigma). The beads were incubated at 4 °C for 3 h and washed twice with ice-cold lysis buffer, three times with the low-salt buffer and once with high-salt buffer. The bound RNAs were purified using TRIzol for the analysis.

### Statistical analysis

All data are presented as mean ± SEM. One way analysis of variance (ANOVA) followed by Dunnett’s test was used for multiple comparisons. A two-tailed value of *P* < 0.05 was considered as statistically significant difference. Statistical analyses were carried out using the GraphPad Prism 5.0 and SPSS 14.0.

## Results

### Identification of lncRNAs that participate as ceRNAs in mesenchymal OvCa

A total of 632 lncRNAs were differentially expressed in both the TCGA and GSE9891 data sets with an FDR < 0.1, and 92.1% of these (582) exhibited the same dysregulation direction (up-regulation or down-regulation) in the iM subtype compared with the iE subtype in both data sets. In addition, 5777 genes were differentially expressed in both the TCGA and GSE9891 data sets with an FDR < 0.1, and 96.5% of these genes (5576 genes) had the same dysregulation direction in the iM subtype compared with the iE subtype in both data sets. Finally, 269 of 377 EMT genes were consistently differentially expressed in both data sets. We next analyzed the correlations among the 269 DE EMT genes and 582 DE lncRNAs identified in the iM OvCa subtype in both data sets using Pearson’s correlation test. Under the constraints of *P* < 0.05 and *r* > 0.4, 114 EMT-lncRNA correlation relationships were identified in the iM OvCa samples in both data sets (Additional file 1: Figure S1). Using information regarding lncRNA-miRNA and miRNA-mRNA interactions, we found that 52 lncRNA-EMT gene pairs shared miRNA binding sites. Of these 52 pairs, 15 had a significantly higher number of common miRNAs than would be expected by chance (*P* < 0.05, hypergeometric test). Figure 1b shows the ceRNA network associated with the iM OvCa subtype. By examining the genomic locations of the lncRNAs and correlated EMT genes, we found that all 15 lncRNA-EMT gene pairs resided on different chromosomes (Fig. 1c).

The article "Systematic analyses reveal long non-coding RNA (PTAF)-mediated promotion of EMT and invasion-metastasis in serous ovarian cancer" was retracted in 2023. Reasons: duplicated images; unreliable results or conclusions.

The lncRNAs and EMT-related genes in Fig. 1b showed significant expression correlations and were significantly up-regulated in iM OvCa samples compared with iE OvCa samples. The SNAI2 gene encodes a transcription factor that represses E-cadherin transcription. E-cadherin is a critical protein that is associated with an epithelial cell phenotype, and E-cadherin down-regulation is believed to be a driver event for EMT involved in cancer invasion and metastasis [32]. We found that SNAI2 was significantly overexpressed in the iM OvCa samples (*P* = 1.59 × 10^− 86^ in TCGA and *P* = 2.07 × 10^− 45^ in GSE9891, t test, Fig. 1d and e) and that OvCa patients with high expression of SNAI2 showed poorer prognosis than those with low SNAI2 expression (*P* = 0.008 in TCGA and *P* = 0.011 in GSE9891, log-rank test, Fig. 1f and g). In the mesenchymal-related ceRNA network, SNAI2 expression was positively correlated with the expression level of the lncRNA LINC00922 in the iM OvCa samples (*P* = 8.73 × 10^− 18^ in TCGA, *P* = 4.58 × 10^− 18^ in GSE9891, Pearson’s correlation test). Among the miRNAs reported to play key roles in the iM subtype of OvCa, miR-25 regulated the largest number of iM-related genes, as reported by Yang et al. [1]. miR-25 was significantly down-regulated in the iM subtype (*P* = 4.28 × 10^− 11^ in TCGA, t test, Fig. 1h). In addition to having binding sites in the 3’-UTRs of predicted targets, miR-25 was also inversely correlated with the expression levels of SNAI2 (*P* = 1.71 × 10^− 9^, Pearson’s correlation test) and the lncRNA LINC00922 (*P* = 0.036, Pearson’s correlation test). LINC00922 was significantly up-regulated in the iM subtype samples compared with the iE subtype samples in the TCGA (*P* = 1.99 × 10^− 15^, t test, Fig. 1i) and GSE9891 (*P* = 9.06 × 10^− 15^, t test, Fig. 1j) data sets. Thus, we hypothesized that LINC00922 up-regulated SNAI2 by competitively binding to miR-25, resulting in induced EMT induction and OvCa cell invasion. For convenience, we have referred to LINC00922 as PTAF (Pro-epithelial-mesenchymal Transition Associated Factor) in this study.

### miR-25 promoted an epithelial phenotype in OvCa cells

To examine the role of the PTAF-miR-25-SNAI2 axis in the progression of OvCa, we first assessed the effect of miR-25 on EMT and OvCa cell migration. We treated SKOV3 and A2780 OvCa cells with TGF-β1, a classical EMT induction factor. As shown in Fig. 2a, miR-25 expression was significantly decreased in the OvCa cells treated with TGF-β1. Next, miR-25 silencing led to the dysregulation of several EMT-associated markers, including decreased CDH1 (E-Cadherin) and increased CDH2 (N-Cadherin), Vimentin, Twist and ZEB1 (Fig. 2b & c). Moreover, a wound-healing assay showed that miR-25 inhibition promoted the migration of both SKOV3 cells and A2780 cells (Fig. 2d). Consistent with these results, a migration assay revealed that miR-25 knockdown induced OvCa cell migration (Fig. 2e).

The article "Systematic analyses reveal long non-coding RNA (PTAF)-mediated promotion of EMT and invasion-metastasis in serous ovarian cancer" was retracted in 2023. Reasons: duplicated images; unreliable results or conclusions.

**Fig. 2:** miR-25 knockdown promotes OvCa cell migration. **a** The expression of miR-25 in OvCa cells after treatment with 10 ng/ml TGF-β1 for 48 h. **b** The mRNA levels of EMT-related markers in SKOV3 cells transfected with a miR-25 inhibitor (AMO-25) or a negative control (NC). **c** Western blotting analysis of epithelial and mesenchymal markers in SKOV3 cells transfected with AMO-25. Wound-healing (**d**) and migration assays (**e**) were used to determine the effect of miR-25 inhibition on OvCa cell migration. *n* = 5 independent experiments. *P < 0.05, **p < 0.01 vs. NC

We further transfected a miR-25 mimic (miR-25) or a scramble negative control (miR-Ctrl) into OvCa cells to determine whether miR-25 overexpression promotes an epithelial phenotype. As illustrated in Additional file 1: Figure S2A & B, forced expression of miR-25 in SKOV3 cells increased the expression of CDH1, decreased the expression of Vimentin at both the mRNA and protein levels, and suppressed other mesenchymal markers, including CDH2, Twist and ZEB1. Furthermore, miR-25 overexpression inhibited wound healing and suppressed migration in both SKOV3 and A2780 cells (Additional file 1: Figure S2C & D).

### miR-25 inhibited TGF-β1-induced EMT in OvCa cells by directly targeting SNAI2

To estimate the potential inhibitory action of miR-25 on EMT, we pre-transfected OvCa cells with miR-25 and then treated them with TGF-β1. As expected, we found that TGF-β1 caused obvious alterations in the expression of EMT-associated genes in SKOV3 cells, whereas pre-transfection with miR-25 rescued the dysregulation of EMT induced by TGF-β1 (Fig. 3a & b). Correspondingly, forced expression of miR-25 in OvCa cells inhibited both TGF-β1-induced wound healing and cell migration (Fig. 3c-f). These results indicate that miR-25 can inhibit TGF-β1-induced EMT and migration in OvCa cells.

**Fig. 3:** Forced expression of miR-25 blunts TGF-β1-induced EMT and migration in OvCa cells. qRT-PCR (**a**) and western blot (**b**) analyses showed the inhibitory effect of miR-25 on EMT in SKOV3 cells treated with TGF-β1. A wound-healing assay displayed the inhibitory effects of miR-25 on TGF-β1-induced migration in SKOV3 cells (**c**) and in A2780 cells (**d**). A migration assay showed that miR-25 attenuated TGF-β1-induced migration in SKOV3 cells (**e**) and A2780 cells (**f**). *n* = 5 independent experiments. *P < 0.05, **P < 0.01

To identify the molecular mechanism underlying the anti-migration effect of miR-25, we constructed pGL3 luciferase expression vectors carrying a fragment of the SNAI2 3′UTR containing either the wild-type (WT) or mutated miR-25 binding site (Fig. 4a). As depicted in Fig. 4b, enhanced expression of miR-25 inhibited the luciferase activity observed after transfection with the WT pGL3-SNAI2, whereas mutating the putative miR-25 binding site (pGL3-SNAI2-Mut) abolished the inhibitory effect of miR-25 on the luciferase activity. Further study showed that miR-25 had no effect on the mRNA expression of SNAI2 (Fig. 4c). However, overexpression of miR-25 decreased the protein level of SNAI2 (Fig. 4d), whereas miR-25 silencing had the opposite effect (Fig. 4e). These results suggest that SNAI2 is a direct target of miR-25 and mediates the effects of miR-25 on EMT and migration in OvCa cells.

The article "Systematic analyses reveal long non-coding RNA (PTAF)-mediated promotion of EMT and invasion-metastasis in serous ovarian cancer" was retracted in 2023. Reasons: duplicated images; unreliable results or conclusions.

**Fig. 4:** SNAI2 is a direct target of miR-25. **a** Sequence alignment showing the complementarity between miR-25 and the human SNAI2 gene. The matched base pairs in the seed region are in red and green. **b** Luciferase reporter activities of chimeric vectors carrying the luciferase gene and a fragment of the SNAI2 3′-UTR containing the wild-type or mutated miR-25 binding site. **c** Overexpression of miR-25 had no effect on the SNAI2 mRNA level. **d** Overexpression of miR-25 repressed the protein expression of SNAI2. **e** Knockdown of miR-25 increased SNAI2 protein expression. *n* = 5 independent experiments. **P < 0.01 vs. miR-Ctrl or NC

### LncRNA PTAF promoted EMT by acting as a ceRNA for miR-25

To determine whether the lncRNA PTAF acts as a ceRNA for miR-25, we first examined the alterations in PTAF expression that occur during EMT. As shown in Fig. 5a & b, PTAF contains a potential miR-25 binding site, and the expression of PTAF was markedly increased in TGF-β1-treated OvCa cells. In addition, we found that PTAF overexpression reduced miR-25 expression (Fig. 5c & d), whereas knocking down PTAF using a specific short hairpin RNA (shRNA) up-regulated miR-25 (Fig. 5e & f). We then constructed a miR-25 sensor luciferase vector containing a perfect miR-25 target site, which was incorporated into the 3’UTR of the luciferase gene. As displayed in Fig. 5g, PTAF overexpression increased the luciferase activity of the miR-25 sensor, whereas PTAF silencing showed the opposite effect, indicating that PTAF binds to miR-25 and relieves the inhibitory effect of miR-25 on its target. Furthermore, forced expression of PTAF alleviated the inhibitory effect of miR-25 on its sensor, whereas a mutated PTAF lacking the binding site for miR-25 failed to do so (Fig. 5h). In addition, biotin-avidin pull-down system was used to examine the direct binding between miR-25 and PTAF. SKOV3 cells were transfected with biotin-tagged miR-Ctrl (Bio-miR-Ctrl) or miR-25 (Bio-miR-25) and then biotin-based pull-down and qRT-PCR assay were performed to test whether miR-25 could pull down PTAF. As shown in Fig. 5i, the introduction of miR-25 caused the enrichment of PTAF, indicating that PTAF can directly bind to miR-25. More importantly, miR-25 overexpression suppressed the luciferase activity of the pGL3-PTAF luciferase vector, whereas it did not exhibit this inhibitory effect on the pGL3-PTAF-Mut luciferase vector (Fig. 5j), in which the miR-25 binding site was mutated (Fig. 5a). Furthermore, overexpression of miR-25 inhibited the expression of PTAF, whereas knockdown of miR-25 had the opposite effect (Fig. 5k & l).

The article "Systematic analyses reveal long non-coding RNA (PTAF)-mediated promotion of EMT and invasion-metastasis in serous ovarian cancer" was retracted in 2023. Reasons: duplicated images; unreliable results or conclusions.

**Fig. 5:** PTAF regulates the expression and activity of miR-25. **a** PTAF contains a sequence domain complementary to the seed motif of miR-25. **b** Up-regulation of PTAF in OvCa cells treated with 10 ng/ml TGF-β1 for 48 h. *n* = 6 independent experiments. **P < 0.01 vs. Control. **c**-**d** Overexpression of PTAF inhibited the expression of miR-25 in SKOV3 cells. *n* = 6 independent experiments. **P < 0.01 vs. pcDNA3.1. **e**-**f** Silencing of PTAF using a specific shRNA up-regulated miR-25 in SKOV3 cells. *n* = 6 independent experiments. *P < 0.05, **P < 0.01 vs. sh-Scramble. **g**-**h** PTAF binds to miR-25 and regulates its activity. *P < 0.05, **P < 0.01. **i** PTAF directly binding to miR-25. SKOV3 cells were transfected with biotin-tagged miR-Ctrl (Bio-miR-Ctrl) or biotin-tagged miR-25 (Bio-miR-25). Forty-eight hours after transfection, the cells were harvested for a biotin-based pull-down assay. PTAF expression levels were analyzed by qRT-PCR. **P < 0.01. **j** Luciferase reporter activities of chimeric vectors carrying the luciferase gene and a fragment of PTAF containing the wild-type (WT) binding site or a mutated binding site for miR-25. **P < 0.01. **k**-**l** qRT-PCR were used to examine the expression of PTAF in SKOV3 cells after overexpression or knockdown of miR-25. *P < 0.05, **P < 0.01. *n* = 6 independent experiments

To validate the role of PTAF in EMT and to determine whether miR-25 mediated this effect, OvCa cells were transfected with PTAF. We found that PTAF overexpression resulted in down-regulation of the epithelial marker CDH1 and up-regulation of mesenchymal markers, indicating the occurrence of EMT (Additional file 1: Figure S3A). Furthermore, forced expression of miR-25 abated the EMT-promoting effect of PTAF, whereas miR-Ctrl failed to do so (Additional file 1: Figure S3A). Enhanced expression of PTAF promoted wound healing and migration in both OVCAR-3 (Fig. 6a & b) and SKOV3 cells (Additional file 1: Figure S3B & C), which could be alleviated by miR-25. In addition, an invasion assay showed that PTAF increased the number of invading OVCAR-3 and SKOV3 cells and that miR-25 attenuated this effect (Fig. 6c**,** Additional file 1: Figure S3D). In contrast, PTAF inhibition almost completely blocked TGF-β1-induced EMT in SKOV3 cells (Additional file 1: Figure S4A). Moreover, PTAF silencing delayed the wound healing, migration and invasion driven by TGF-β1 in OVCAR-3 (Fig. 6d-f) and SKOV3 cells (Additional file 1: Figure S4B-D). More importantly, miR-25 knockdown markedly attenuated the inhibitory effect of PTAF silencing on TGF-β1-induced migration and invasion in OvCa cells (Fig. 6d-f, Additional file 1: Figure S4). The above results suggest that miR-25 mediates the EMT-promoting effect of the lncRNA PTAF.

The article "Systematic analyses reveal long non-coding RNA (PTAF)-mediated promotion of EMT and invasion-metastasis in serous ovarian cancer" was retracted in 2023. Reasons: duplicated images; unreliable results or conclusions.

**Fig. 6:** PTAF overexpression leads to OVCAR-3 cell migration and invasion by regulating miR-25. Wound-healing **a** and migration assays **b** showed that PTAF promoted OVCAR-3 cell migration, which was inhibited by forced expression of miR-25. *n* = 5 independent experiments. *P < 0.05*,* **P < 0.01. **c** A Transwell invasion assay showed that PTAF promoted OVCAR-3 cell invasion by regulating miR-25. *n* = 5 independent experiments. **P < 0.01. Wound-healing **d** and migration assays **e** showed that silencing of PTAF inhibited TGF-β1-driven migration in OVCAR-3 cells, which was abated by miR-25 knockdown. *n* = 5 independent experiments. *P < 0.05*,* **P < 0.01. **f** A Transwell invasion assay showed that knockdown of PTAF inhibited TGF-β1-induced OVCAR-3 cell invasion. *n* = 5 independent experiments. *P < 0.05*,* **P < 0.01

### Silencing PTAF inhibited tumor progression and metastasis in an orthotopic mouse model of OvCa

To validate the role of PTAF in vivo, we generated luciferase-labeled SKOV3 cells and intraperitoneally injected these cells into nu/nu mice to establish an OvCa orthotopic mouse model. Bioluminescence images showed that PTAF overexpression promoted tumor growth (Fig. 7a & b) and liver metastasis in vivo (Fig. 7c). Moreover, forced expression of PTAF strikingly increased the number of tumor modules and tumor weight compared with empty pcDNA3.1 (Fig. 7d). Meanwhile, immunohistochemical staining demonstrated that mice injected with PTAF-overexpressing cells exhibited lower E-cadherin expression and higher SNAI2 expression than mice injected with cells overexpressing empty pcDNA3.1 (Fig. 7e).

The article "Systematic analyses reveal long non-coding RNA (PTAF)-mediated promotion of EMT and invasion-metastasis in serous ovarian cancer" was retracted in 2023. Reasons: duplicated images; unreliable results or conclusions.

**Fig. 7:** PTAF silencing inhibits tumor progression in an orthotopic mouse model of OvCa. **a** Representative bioluminescence images of mice injected intraperitoneally with SKOV3 OvCa cells expressing either PTAF or empty pcDNA3.1 (*n* = 10 in each group). **b** More tumor masses (yellow arrows) were formed by SKOV3-PTAF cells than by SKOV3-pcDNA3.1 cells. **c** Mice injected with SKOV3-PTAF cells showed liver metastases. **d** Representative images of tumor nodules and quantification of tumor nodules and tumor weights in mice injected intraperitoneally with SKOV3 OvCa cells expressing either PTAF or empty pcDNA3.1 (*n* = 10 in each group). **P < 0.01 vs. pcDNA3.1. **e** SKOV3-ip tumor samples from mice injected with cells expressing PTAF or empty pcDNA3.1 were immunohistochemically stained for E-cadherin and SNAI2. *P < 0.05 vs. pcDNA3.1. **f** Representative bioluminescence images in sh-Scramble- and sh-PTAF-treated mice (*n* = 10 in each group) that were injected intraperitoneally with SKOV3 OvCa cells. **g** Fewer tumor masses (yellow arrows) were formed in the mice treated with sh-PTAF than in those treated with sh-Scramble. **h** Mice injected with sh-Scramble showed liver metastases, whereas very little metastasis was observed in mice injected with sh-PTAF. **i** Representative images of tumor nodules and quantification of tumor nodules and tumor weights in sh-Scramble- and sh-PTAF-treated mice injected with SKOV3 cells (*n* = 10 for each group). **P < 0.01 vs. sh-Scramble. **j** SKOV3-ip tumor samples from sh-Scramble- and sh-PTAF-treated mice were immunohistochemically stained for E-cadherin and SNAI2. *P < 0.05 vs. sh-Scramble. Scale bars, 100X = 100 μm; 400X = 20 μm

Finally, to determine the therapeutic effect of PTAF suppression, we generated the stable PTAF knockdown or overexpression luciferase-labeled SKOV3 cells and then intraperitoneal injected the cells into female BALB/c nude mice to establish the orthotopic mouse model of OvCa. Contrary to the above results, PTAF knockdown inhibited the growth (Fig. 7f & g) liver metastasis of the SKOV3 cells (Fig. 7h). More excitingly, silencing PTAF reduced the number of tumor nodules and the tumor weight (Fig. 7i) and resulted in increased E-cadherin expression and decreased SNAI2 expression compared with mice injected with a lentivirus carrying an sh-Scramble construct (Fig. 7j). These results showed that PTAF may be a potential target in OvCa treatment.

The article "Systematic analyses reveal long non-coding RNA (PTAF)-mediated promotion of EMT and invasion-metastasis in serous ovarian cancer" was retracted in 2023. Reasons: duplicated images; unreliable results or conclusions.

### Correlation between the lncRNA PTAF and EMT markers in OvCa

To further evaluate the association between the lncRNA PTAF and EMT in OvCa, we acquired a cohort of 49 clinically annotated OvCa tumor samples from the Second Affiliated Hospital of Harbin Medical University. The expression of PTAF was measured using ISH on formaldehyde-fixed, paraffin-embedded tissue sections from these patients. We also performed immunohistochemical staining for E-cadherin and SNAI2 and used quantitative RT-PCR analysis to measure miR-25 expression in frozen tissues. We found that tumors with low PTAF expression exhibited more epithelial characteristics, whereas those with high PTAF expression exhibited a more mesenchymal phenotype (Fig. 8a). Moreover, PTAF expression was inversely correlated with E-cadherin protein expression and positively correlated with SNAI2 expression (Fig. 8b). In addition, PTAF expression was inversely correlated with miR-25 expression (Fig. 8c). The mesenchymal OvCa patients in the TCGA dataset with high PTAF expression showed a poorer prognosis than those with low PTAF expression (*P* = 0.043, log-rank test, Fig. 8d).

**Fig. 8:** Correlation between PTAF and E-cadherin, SNAI2 and miR-25 expression in serous OvCa cohorts. **a** Representative images of in situ hybridization staining for PTAF and immunohistochemical staining for E-cadherin and SNAI2 in low and high PTAF expression cases. PTAF expression was stratified by using the average PTAF PCR expression as a threshold. **b** Bar charts show the association between PTAF expression and E-cadherin and SNAI2 expression. **c** The association between PTAF expression and miR-25 expression, as measured by qRT-PCR. **d** Kaplan-Meier overall survival curves for the mesenchymal OvCa patients with high and low expression of PTAF in the TCGA data set. **e** Up-regulation of the lncRNA PTAF induced SNAI2 expression by competitively binding miR-25, which promoted OvCa cell EMT and invasion. **P < 0.01 vs. PTAF Low. Scale bars, 100X = 100 μm; 400X = 20 μm

## Discussion

In this study, we present evidence from systems-based miRNA, lncRNA and mRNA analyses of large-scale OvCa data sets along with in vitro and in vivo experiments showing that the lncRNA PTAF is a key regulator of EMT and promotes the OvCa invasion-metastasis cascade. Up-regulation of PTAF induced elevated expression of SNAI2, a transcriptional repressor of E-cadherin, by competitively binding miR-25, which resulted in the promotion of OvCa cell EMT and invasion (Fig. 8e). We demonstrated that miR-25 inhibits the mesenchymal phenotype and TGF-β1-induced EMT by directly targeting SNAI2. We established the importance of PTAF-miR-25-SNAI2 in the EMT process by demonstrating the positive correlation PTAF and SNAI2 expression and the inverse correlations between miR-25 and PTAF expression and miR-25 and SNAI2 expression in iM OvCa samples. Our findings not only suggest the important role of lncRNAs as miRNA sponges in the regulation of EMT progression in OvCa but also underscore the potential of the lncRNA PTAF as a target for inhibiting EMT in OvCa.

The article "Systematic analyses reveal long non-coding RNA (PTAF)-mediated promotion of EMT and invasion-metastasis in serous ovarian cancer" was retracted in 2023. Reasons: duplicated images; unreliable results or conclusions.

The information from high-throughput studies, such as that deposited in TCGA, have allowed comprehensive investigations of EMT mechanisms using integrated analyses of multi-dimensional cancer case data [33]. Our integrated approach revealed an activated ceRNA regulatory network involved in the EMT process in iM OvCa patients (Fig. 1b). Yang et al. described a miRNA regulatory network consisting of eight key miRNAs in the iM subtype of OvCa cases. Among the eight miRNAs, miR-25, miR-182, miR-128, miR-101, miR-141, and miR-200a were found in our ceRNA regulatory network. Two other miRNAs, miR-506 and miR-29c, were not included in our regulatory network because of the statistical controls used during the selection of ceRNAs. Among the six miRNAs in the iM-related ceRNA regulatory network, miR-25 regulates the largest number of targets in the miRNA regulatory network, as reported by Yang et al. However, the role of miR-25 in EMT and OvCa remains unclear [15]. As previously reported [34, 35], we also found that miR-25 was significantly up-regulated in OvCa patients compared with normal ovarian tissue (*P* = 9.05 × 10^− 7^, t test). Interestingly, miR-25 was significantly down-regulated in patients with the iM subtype of OvCa compared with patients with the iE subtype (*P* = 4.28 × 10^− 11^, t test). By analyzing miRNA-target interactions and expression profiles, we found that miR-25 not only had binding sites within SNAI2, a key TF regulating EMT, and PTAF but also had an inverse expression relationship with both SNAI2 and PTAF. Thus, we narrowed our focus to the functional investigation of the role of PTAF-miR-25-SNAI2 in EMT in iM OvCa patients. According to the lncRNA-EMT gene correlation network (Additional file 1: Figure S1), PTAF expression is also significantly correlated with the gene *MMP13*, *FN1*, *FGF1*, *MMP2*, *PDPN*, *POSTN*, *VCAN*, and *LOXL2* in mesenchymal OvCa, which indicates that PTAF may promote EMT in OvCa by regulating these EMT-related genes.

Notably, in this study, we also revealed many other key ceRNA relationships, such as the relationship between the lncRNA HAND2-AS1 and ZEB1, another key TF in EMT. Both HAND2-AS1 and ZEB1 have binding sites with the known EMT-related miRNAs miR-200a, miR-141, and miR-101. The lncRNA HAND2-AS1 has been reported to be associated with metastasis in hepatocellular carcinoma [36]. These newly identified ceRNA relationships may have potential roles in the iM subtype of OvCa and warrant further study.

The article "Systematic analyses reveal long non-coding RNA (PTAF)-mediated promotion of EMT and invasion-metastasis in serous ovarian cancer" was retracted in 2023. Reasons: duplicated images; unreliable results or conclusions.

## Conclusion

In summary, our integrated analysis uncovered a ceRNA regulatory network for the mesenchymal subtype of serous OvCa and highlighted the important role of the lncRNA PTAF in promoting EMT in OvCa by regulating SNAI2 expression through miR-25. The findings of our study have significant implications regarding our understanding of OvCa metastasis. As direct targets of the lncRNA PTAF, miR-25 and SNAI2 mediated its role in local invasion and metastasis, respectively. The effects of PTAF on the invasion-metastasis cascade suggest that it could be an effective target for anti-metastasis therapies in OvCa.

## Additional file

Additional file 1: **Table S1.** Statistics of datasets. **Figure S1.** LncRNA-EMT gene correlation network in mesenchymal ovarian cancer. Nodes marked by rounded rectangle and ellipse denote lncRNA and EMT gene, respectively. Nodes with blue or green color represent lncRNA or EMT genes are significantly up-regulated in mesenchymal OvCa compared with epithelial OvCa. The edges represent the significant correlation between lncRNAs and EMT genes. **Figure S2.** Overexpression of miR-25 in OvCa cells promotes epithelial phenotype. (A) The mRNA levels of EMT-related markers in SKOV3 cells transfected with miR-25 or control miRNA (miR-Ctrl). (B) Quantification of E-cadherin and Vimentin in SKOV3 cells transfected with miR-25 or control miRNA (miR-Ctrl). Wound healing assay (C) and migration assay (D) determined the effect of miR-25 on cell migration in OvCa cells. *n* = 5 independent experiments. *p < 0.05, **p < 0.01 vs. miR-Ctrl. **Figure S3.** PTAF promoted migration in SKOV3 cells. (A) Overexpression of PTAF induced EMT by regulating miR-25 in SKOV3 cells, as measured by qRT-PCR. *n* = 6 independent experiments. *P < 0.05. Wound-healing (B) and migration assays (C) showed that PTAF promoted SKOV3 cell migration, which was inhibited by forced expression of miR-25. *n* = 5 independent experiments. *P < 0.05, **P < 0.01. (D) A Transwell invasion assay showed that PTAF promoted SKOV3 cell invasion by egulating miR-25. *n* = 5 independent experiments. **P < 0.01. **Figure S4.** Silencing of PTAF inhibited TGF-driven migration in SKOV3 cells. (A) Knockdown of PTAF attenuated TGF-β1-induced EMT in SKOV3 cells, which could be alleviated by miR-25 inhibition. *n* = 6 independent experiments. *P < 0.05. Wound-healing (B) and migration assays (C) showed that silencing of PTAF inhibited TGF-β1-driven migration in SKOV3 cells, which was abated by miR-25 knockdown. *n* = 5 independent experiments. *P < 0.05, **P < 0.01. (D) A Transwell invasion assay showed that knockdown of PTAF inhibited TGF-β1-induced SKOV3 cell invasion. *n* = 5 independent experiments. **P < 0.01. (DOC 13561 kb)

The article "Systematic analyses reveal long non-coding RNA (PTAF)-mediated promotion of EMT and invasion-metastasis in serous ovarian cancer" was retracted in 2023. Reasons: duplicated images; unreliable results or conclusions.

## Abbreviations

BH: Benjamini-Hochberg
ceRNA: Competing endogenous RNA
DE: Differentially expressed
EMT: Epithelial-Mesenchymal Transition
FDR: False discovery rate
iE: Integrated epithelial
IHC: Immunohistochemistry
iM: Integrated mesenchymal
ISH: In situ hybrization
LncRNAs: Long non-coding RNAs
OvCa: Ovarian cancer
shRNA: Short hairpin RNA
WT: Wide type
